This article has been retracted.

# Santacruzamate A Ameliorates AD-Like Pathology by Enhancing ER Stress Tolerance Through Regulating the Functions of KDELR and Mia40-ALR *in vivo* and *in vitro*

**DOI:** 10.3389/fncel.2019.00061

**Published:** 2019-03-04

**Authors:** Lei Chen, Yue-cheng Liu, Hui Tan, Yuan Zhang, Ji Xu, Wen-lan Liu, Zong-yang Li, Wei-ping Li

**Affiliations:** ^1^Shenzhen Key Laboratory of Neurosurgery, Brain Center, Shenzhen Second People’s Hospital, Shenzhen University 1st Affiliated Hospital, Shenzhen, China; ^2^Guangzhou Medical University, Guangzhou, China

**Keywords:** santacruzamate A, Aβ_25–35_, APPswe/PS1dE9 mice, KDEL receptor, Mia40

## Abstract

Aggregated amyloid-β protein (Aβ) and Aβ-induced neuronal apoptosis have been implicated as critical factors in the pathophysiology of Alzheimer’s disease (AD). Certain preclinical results have indicated that the increased accumulation of protein aggregates in AD-affected neurons activates the unfolded protein response (UPR), a pathological phenomenon, which predominantly mediates the aberrant endoplasmic reticulum (ER) stress and apoptotic cascades in neuronal cells. In the present study, we confirmed that Santacruzamate A (STA, a natural product isolated from a Panamanian marine cyanobacterium) attenuates Aβ protein fragment 25–35 (Aβ_25–35_)-induced toxicity in PC12 cells and rescues cognitive deficits in APPswe/PS1dE9 mice by enhancing ER stress tolerance. We first demonstrated the anti-apoptotic effects of STA by evaluating caspase-3 activity, annexin V/propidium iodide (PI) staining, and terminal deoxynucleotidyl transferase dUTP nick end labeling staining. Behavioral testing of STA-treated APPswe/PS1dE9 mice showed that the pronounced memory impairments were ameliorated and that the consolidated memories were stably maintained over a 2-week period. The mechanistic studies provided evidence that STA inhibited Aβ_25–35_-induced UPR and ER stress by regulating the ER retention signal (KDEL) receptor, which reinforced the retention of resident chaperones in the ER lumen. Furthermore, STA regulated the expression of the mitochondrial intermembrane space assembly protein 40 (Mia40) and augmenter of liver regeneration (ALR), which ultimately attenuated the mitochondrial fission and apoptosis pathways. Together, our present findings suggest that the KDEL receptor and Mia40-ALR play a role in mitigating Aβ_25–35_-induced neurotoxicity, which might in turn positively regulate learning and memory. These observations support that STA may be a promising agent for reversing the progression of AD.

## Introduction

Alzheimer’s disease (AD) is a slow and progressive age-related neurodegenerative disease that is characterized by debilitating memory impairments, as well as by the progressive accumulation of extensive extracellular amyloid-β protein (Aβ) plaques and intracellular neurofibrillary tangles (Mullan et al., 1992). Several studies have shown that soluble oligomers of Aβ are sufficient to cause structural and functional changes to neurons (Hardy and Selkoe, 2002). As the disease progresses, elevated levels of Aβ are believed to induce extensive neuronal loss and cognitive function deterioration, which are hypothesized to contribute to the neurodegeneration and memory impairments that are associated with AD (Butterfield et al., 2002). Therefore, any substance that can prevent Aβ-induced neuronal apoptosis may be useful as a new therapeutic agent for the treatment or prevention of AD.

Long-term failure of quality control in neuronal cells may cause protein aggregation, leading to neurodegeneration (Ogen-Shtern et al., 2016). As a neurotoxin, the pathological concentration of Aβ has been demonstrated to lead to an excess of misfolded proteins, which further provokes prolonged endoplasmic reticulum (ER) stress until neuronal death occurs (Chan et al., 2004; Katayama et al., 2004). The ER is a vast membranous subcellular compartment that is responsible for the maturation, folding, and trafficking of a wide range of proteins (Brodsky and Skach, 2011). Therefore, Aβ aggregation compromises the folding and maturation of newly synthesized proteins, ultimately causing ER stress (Costa et al., 2010). To manage ER stress, an elaborate adaptive process known as the unfolded protein response (UPR) is stimulated to augment protein folding and restore ER homeostasis (Smith et al., 2011). However, in cases of aggressive or persistent Aβ deposition and impairment, if the accumulated misfolded proteins cannot be cleared to restore homeostasis, an unmitigated UPR would cause protracted ER stress, which could be lethal and trigger apoptotic cascades (Yoshida et al., 2001). In addition, an increasing body of evidence has suggested that mitochondria cooperate to produce Aβ-induced ER stress and a cell death signal. That is, when functional mitochondria are in the presence of the Aβ peptide, this may lead to ER stress and ER calcium release, activating an ER-stress mediated apoptotic pathway that involves the translocation of Bax to the mitochondria, loss of the mitochondrial membrane potential (MMP), cytochrome c release, and activation of caspase-9 and caspase-3, finally leading to apoptotic cell death. Although the molecular mechanisms underlying these processes are not completely understood, the structural and functional networks of the mitochondria and ER seem to be essential in determining the cell fate under Aβ-related pathophysiological conditions (Costa et al., 2010, 2012). Therefore, attenuating Aβ-induced ER stress and blocking the concomitant mitochondrial apoptotic pathway might be a promising avenue for treating the Aβ-related neuronal loss and memory impairments of AD.

Prior research has revealed that the KDEL receptor (KDELR) is involved in ER stress and ER quality control by recognising the C-terminal motif (Lys-Asp-Glu-Leu sequence) of the ER-resident chaperones in the post-ER compartment (Yamamoto et al., 2003) and returning them to the ER lumina (Capitani and Sallese, 2009). Importantly, ER-retained chaperones, such as protein disulfide isomerase (PDI) and glucose regulated protein 78 and 94 (GRP78 and GRP94), are localized to the ER (Lewis and Pelham, 1992) and are responsible for the folding and degradation of newly synthesized or misfolded proteins (Butler et al., 2011). Under cellular stress circumstances, regulation of the transport and retrieval system of essential chaperones promotes the retrieval and return of misfolded proteins back to the ER for refolding or ER-associated degradation, and as such makes a vital contribution to ER protein quality control. The KDELR has also been shown to participate in the degradation of misfolded neurodegenerative disease-related proteins (Wang et al., 2011). Therefore, the KDELR may play crucial roles in Aβ-induced ER stress and in the concomitant apoptotic signaling pathway by regulating ER-retained chaperone transport and misfolded protein modification. However, studies investigating the involvement of the KDELR in the Aβ-induced ER stress and apoptosis of AD are needed. Further, it remains unknown whether agents targeting KDELR or related mitochondrial elements could serve as treatments for AD.

In the present study, we confirmed the neuroprotective effects of a carbamate derivative, Santacruzamate A (STA, a natural product isolated from a Panamanian marine cyanobacterium), against Aβ_25–35_-induced toxicity in PC12 cells and identified the restorative effects of STA on the memory impairments in APPswe/PS1dE9 mice *via* behavioral testing. The mechanistic studies we performed demonstrated that STA inhibited harmful Aβ_25–35_-induced ER stress and blocked Aβ_25–35_-induced ER chaperone translocation to the mitochondria by activating the KDELR, reversing the function of mitochondrial intermembrane space assembly protein 40 (Mia40)-augmenter of liver regeneration (ALR), restoring the mitochondrial intermembrane space assembly, and attenuating the mitochondrial fission pathway. The findings of this study shed new light on the pharmacological mechanisms and consequences of using this type of carbamate derivative as a treatment for AD and reveal that STA might be a candidate therapeutic compound for some neurodegenerative disorders. In particular, our data suggest that STA modulates the functions of the KDELR and Mia40-ALR, which might be appropriate synergistic targets for suppressing Aβ-induced ER stress and the associated mitochondrial cell death pathways.

## Materials and Methods

### Reagents and Cell Treatment

Amyloid β protein fragment 25–35 (Aβ_25–35_) was purchased from Sigma-Aldrich (St. Louis, MO, USA), and was dissolved in sterile saline and incubated at 37°C for 7 days to allow for fibril formation as described previously (Giovannelli et al., 1995). The fibril-like structures and globular aggregates were confirmed microscopically. STA (purity≥98.0%) was purchased from Selleck Chemicals (TX, USA). Fetal bovine serum (FBS), heat-inactivated horse serum, Dulbecco’s Modified Eagle Medium (DMEM), DMEM/F12, L-glutamine, penicillin and streptomycin were purchased from Gibco (NY, USA). PC12 and SH-SY5Y neuroblastoma cells were obtained from the Chinese Academy of Medical Sciences and were cultured *in vitro* as described previously (Li et al., 2016b). Cells in the exponential growth phase were used for all experiments. To study the anti-apoptotic effects of STA, cells were divided into the untreated control, STA alone, Aβ_25–35_ (25 μM), and Aβ_25–35_ (25 μM) plus STA groups. The STA was first dissolved in dimethyl sulfoxide (DMSO) at a concentration of 10 mM and then in Dulbecco’s Modified Eagle’s medium immediately before use. Final preparations contained less than 0.1% (v/v) DMSO, and DMSO was used as the vehicle control medium. Cells were pre-incubated with different concentrations of STA for 4 h and subsequently co-cultured with 25 μM of a prepared Aβ_25–35_ peptide for an additional 8 h for the mechanistic investigation or 24 h for the pharmacodynamics analysis.

### Cell Viability and Apoptosis Assays

Cell viability was evaluated with the Cell Counting Kit-8 (CCK-8) as described previously (Li et al., 2016b). The cell damage was determined by the release of lactate dehydrogenase (LDH) into the incubation medium using the assay kit (Nanjing Jiancheng Bioengineering Institute, China) according to the manufacturer’s instructions. Briefly, after the treatment, the cells in 6-well plate were centrifuged at 1,000 *g* for 4 min, 1 mL culture supernatants were collected from each well; 3.4 mL reaction buffer supplied in the kit was then added. 30 min after mixing at room temperature, the release of LDH was assessed using a microplate reader at a test wavelength of 340 nm and expressed as a percentage (%) of total LDH activity (LDH in the medium + LDH in the cell), according to the equation % LDH released = (LDH activity in the medium/total LDH activity) × 100. Each experiment was performed for four times. The caspase-3 activity determination was detected using the assay kit (Merck-Millipore, USA). Cells were harvested by centrifugation and the media removed. A volume of 50 μl of 10 μM substrate solution (PhiPhilux is a unique class of substrates for caspase-3) was added to the cell pellet (1 × 10^5^ cells per sample); the cells were not vortex mixed. Cells were incubated at 37°C for 60 min, then washed once by adding 1 ml of ice-cold PBS and were re-suspended in 1 ml fresh PBS. Cells were analyzed with a flow cytometer (Becton-Dickinson) equipped with an argon ion laser at 488 nm wavelength. Caspase-3 activity was determined and analyzed. The DNA fragmentation of apoptotic PC12 cells was detected using a terminal deoxynucleotidyl transferase-mediated biotinylated UTP nick end labeling (TUNEL) kit (Roche Diagnostics Corp., IN, USA). The cells were cultured on coverslips for 24 h. At the end of the drug treatment, the cells were fixed by incubation in a 10% neutral buffered formalin solution for 30 min at room temperature. Next, the cells were incubated with a methanol solution containing 0.3% H_2_O_2_ for 30 min at room temperature and then incubated with a permeabilizing solution (0.1% sodium citrate and 0.1% Triton X-100) for 2 min at 4°C. The cells were incubated with the TUNEL reaction mixture for 60 min at 37°C and visualized by inverted fluorescence microscopy (Leica, Germany). The TUNEL-positive nuclei of four non-overlapping fields per coverslip were counted, and these counts were converted to percentages by comparing the TUNEL-positive counts to the total numbers of cell nuclei, as determined by DAPI counterstaining. Furthermore, cell apoptosis was determined using annexin V/propidium iodide (PI) assay as described previously (Li et al., 2016a).

### Electrophysiological Recordings

All recordings were made at 37°C using an EPC10 patch-clamp amplifier (HEKA Electronic, Germany) and PULSE software (HEKA). A whole-cell configuration of the patch clamp technique was used throughout. The acquisition rate was 10 kHz and signals were filtered at 2.5 kHz. Patch electrodes were pulled with a horizontal micropipette puller (P-97 Sutter Instruments, Novato, CA, USA) and fire polished. The recording electrodes had tip resistance of 2–4 MΩ when filled with the pipette solution, which contained (in mM) 135 CsCl; 3 MgCl_2_; 10 EGTA; 10 HEPES; 3 Mg-ATP; 0.6 GTP (pH 7.4 adjusted with CsOH). The external solution contained (in mM) 150 TEA-Cl; 2 CaCl_2_; 10 HEPES; 10 glucose (pH 7.4 adjusted with CsOH). L-type Ca^2+^ currents, that had been verified by adding 5 μM Nifedipine, were measured by 150 ms square voltage pulses to 10 mV from a holding potential of -50 mV. A low-profile perfusion chamber fed by a gravity perfusion system was used for solution exchange.

### Purification of Subcellular Fractionation

Cell pellets were gently resuspended in cytoplasmic buffer (10 mM Hepes, pH 7.4; 1.5 mM MgCl_2_, 10 mM KCl, 0.5 mM DTT, 10 mM Na_2_MoO_4_, 2 mM PMSF, 20 mg/ml aprotinin, 0.1% NP-40; 25 mM NaF, and 0.2 mM Na_3_VO_4_) and kept on ice for 10 min before centrifugation at 900 *g* for 10 min. The nuclear pellets were processed as described below. The cytoplasmic supernatant was recentrifuged at 900 *g* to ensure complete removal of nuclear material. The resulting supernatant was centrifuged at 10,000 *g* for 30 min. The cytosolic supernatant was processed for Western blot by adding protein sample buffer (PSB) 4.5. The mitochondrial pellet was washed with cytoplasmic buffer, recentrifuged at 10,000 *g*, and dissolved in PSB 1.5. The nuclear pellet was washed with cytoplasmic buffer and recentrifuged at 900 *g* before their extraction in nuclear buffer (20 mM Hepes, pH 7.4, 1.5 mM MgCl_2_, 420 mM NaCl, 25% glycerol (vol/vol), 0.2 mM EDTA, 0.5 mM DTT, 10 mM Na_2_MoO_4_, 2 mM PMSF, 20 mg/ml aprotinin, 25 mM NaF, and 0.2 mM Na_3_VO_4_). The Oncogene cytosol/mitochondria fractionation kit (QIA88; Onco-gene Research Products) was used according to the manufacturer’s instructions.

### Immunoblot Analyses and Immunoprecipitates

At the end of treatment, the cells were harvested and washed once with PBS, and the cells used for other quantities of proteins were lysed in a cell lysis buffer containing 1% phenyl methyl sulfonyl fluoride (PMSF). The whole cell lysates were centrifuged at 12,000 rpm for 5 min at 4°C, and the supernatants were collected. Protein concentration was determined by bicinchoninic acid assay. Equal amounts of protein (10 μg) were separated by electrophoresis on 10% sodium dodecyl sulfate polyacrylamide gels and transferred onto nitrocellulose membranes. These membranes were incubated with 5% (w/v) non-fat milk powder in Tris-buffered saline containing 0.1% (v/v) Tween-20 (TBST) for 40 min to block nonspecific binding sites. The membranes were then incubated overnight at 4°C with the primary antibodies. After washing with TBST, the membranes were incubated for 1 h at room temperature with the secondary antibodies. After rewashing with TBST, the bands were developed by enhanced chemiluminescence with primary antibodies obtained from the following sources: anti-GAPDH, anti-Tom40, anti-Tim23, anti-Tim17, anti-COX17, anti-Cytochrome C, anti-caspase-9, anti-caspase-12, anti-Cytochrome, anti-VDAC protein, anti-Histone H2B, anti-α-tubulin, anti-PDI, anti-IREα, anti-p-IREα, anti-eIF2α, anti-p-eIF2α, anti-Mia40, anti-ALR, anti-Fis1, anti-Mff, anti-MiD49, anti-PERK and anti-p-PERK (Abcam); anti-KDEL receptor, anti-GADD153, anti-ATF4, anti-Bax, anti-AIF, anti-Smac and anti-GRP78 (Santa Cruz, CA, USA); anti-COX6B were purchased from Sigma-Aldrich (Sigma, CA, USA). The secondary peroxidase-conjugated antibodies were purchased from Cell Signalling Technology (Beverly, MA, USA). Immunoprecipitation of GRP78 and PERK were carried out using specific-antibodies and immunoblotted with anti-GRP78 or anti-PERK antibodies, respectively. Class-specific IgG antibodies were used as controls in the immunoprecipitation experiments. Cells were lysed with lysis buffer (50 mM Tris, pH 7.4, 150 mM NaCl, 1 mM EDTA, 1% Nonidet P-40, and protease inhibitor cocktail) on ice for 1 h. After centrifuging at 12,000 rpm for 20 min, the lysates (1–2 mg) were incubated with an anti-GRP78 antibody overnight at 48°C on a rotary wheel. Immunoprecipitates were collected by incubating with 20 μl of protein A magnetic beads (Millipore) for 2 h at 4°C. Then, the immunoprecipitates were washed five times with PBS, resuspended and boiled in 30 ml of sample loading buffer. The samples were subjected to electrophoresis, and GRP78 and PERK were detected by immunoblotting. Horizontal scanning densitometry was conducted on blots using Adobe PhotoShop (Adobe Systems, Inc.). Images were acquired using a Leica fluorescence microscope (Leica, Germany).

### Immunofluorescence Microscopy

For immunofluorescence analysis, cells growing on glass coverslips were washed with PBS and then fixed with 4% (w/v) paraformaldehyde for 20 min at 37°C. The cells were washed with PBS, permeabilized with 0.1% (v/v) Triton X-100 for 1 h, and blocked for 30 min in medium containing serum. After an additional wash with PBS, immunostaining was performed by incubating the cells with primary antibodies for 2 h at room temperature (25°C). Primary antibodies were diluted in 0.1% (v/v) Triton X-100, 0.2% (w/v) BSA, 0.5 mM PMSF and 1 mM dithiothreitol in PBS. After washing with PBS, the bound primary antibodies were detected using FITC-conjugated goat anti-rabbit antibodies, Cy5-conjugated goat anti-mouse antibodies or Cy5-conjugated donkey anti-rabbit antibodies for 2 h at room temperature. Images were acquired using a Leica fluorescence microscope (Leica, Germany).

### Measurement of Mitochondrial Permeability Transition Pore (mPTP) Opening and Mitochondrial Membrane Potentials (MMPs)

The opening of the mitochondrial permeability transition pore (mPTP) in treated PC12 cells was determined using the calcein-cobalt quenching Detection Kit (Genmed Scientifics, Inc.). All procedures completely complied with the manufacturer’s instructions. The cells were cultured in 24-well plates. After the indicated treatments, PC12 cells were loaded with calcein dye and in the presence of cobalt chloride (CoCl_2_ 1 mmol/L) at 37°C for 30 min. Images were acquired using a Leica fluorescence microscope (Leica, Germany) with excitation and emission wavelengths of 488 and 505 nm, respectively. The opening of mPTP in each group was calculated as the fluorescence intensity. The opening of mPTP was analyzed using a fluorescence microplate reader after calcein-cobalt staining. The results are expressed as a percentage of control. 5,5’,6,6’-tetrachloro-1,1’,3,3’-tetraethylbenzimidazolyl-carbocyanine iodide (JC-1, Invitrogen, Eugene, OR, USA) was used to determine the changes in MMP in the treated PC12 cells. Briefly, the cells were suspended in warm medium at approximately 1 × 106 cells/ml and then incubated with JC-1 (2 mM final concentration) for 30 min in the dark. After incubation, the cells were washed twice with PBS and visualized using a fluorescence microscope (Leica, Germany). Monomeric JC-1 green fluorescence emission and aggregate JC-1 red fluorescence emission were measured on a microplate reader. The MMP of the PC12 cells in each treatment group were calculated as the ratios of red to green fluorescence.

### Transfections

PC12 cells were transiently transfected according to the instructions of the manufacturer using Lipofectamine and Plus Reagent (Invitrogen) with plasmids containing scrambled oligonucleotide (control siRNA) or siRNA. The KDELR siRNA with the sequences sense 5’-CCACGGUCUGGUUGAUUUATT-3’ and antisense 5’-UAAAUCAACCAGACCGUGGTG-3’ and scrambled control siRNA were designed and synthesized by Gene Pharma (Beijing, China). siRNA was transfected into cells using RNAiMAX lipofectamine (Invitrogen) in Opti-MEM reduced serum medium (Invitrogen). siRNA was incubated with RNAiMAX for 30 min at room temperature prior to transfection, and the targeted protein expression levels were silenced during a 2-day incubation.

### Animal Treatments and Biochemical Evaluation

All animal procedures were performed in accordance with the National Institutes of Health Guidelines on the Use and Care of Animals and approved by the Institutional Animal Experiment Committee of Shenzhen Second People’s Hospital. Healthy male 6-month-old double-transgenic APPswe/PS1dE9 (APP/PS1) and wild type (WT) littermates were obtained from the Institute of Laboratory Animal Science, Chinese Academy of Medical Science (Beijing, China). After 7 days of habituation, the animals were divided into four groups, APP/PS1 mice (*n* = 60) were randomly assigned into vehicle-treated group (*n* = 20), STA (*n* = 20, 5 mg/kg/day, by gavage), STA (*n* = 20, 10 mg/kg/day, by gavage), and WT littermates (*n* = 20, given the same volume of vehicle and used as control) for a period of 8 weeks. WT and APP/PS1 mice were administered with saline. Body weight and physical performance of all mice were measured. There were no significant differences among groups before 1d and after 1d of medication. Locomotive activities of mice were tested in open-field on the first day of behavioral test. Morris water maze (MWM) tests were carried out on day 2 to day 8 and day 23 to day 25; step-down passive avoidance tests were valued on day 15 to day 16 and day 28, respectively. After behavioral measurements, mice (*n* = 8 per group) were sacrificed by decapitation; the brain tissues were quickly removed, washed with cold saline solution, followed by 50 mM Tris-HCl buffer (pH 7.4), and weighed. Then, it was placed into a glass bottle, labeled, and stored in a deep freezer (−25°C) until processing (maximum 10 h). The tissues were homogenized in four volumes of ice-cold Tris-HCl buffer (50 mM, pH 7.4) using a glass Teflon homogenizer (Elektro-crafts, Mumbai) for 2 min at 5,000 rpm after cutting it into small pieces. The homogenate was then centrifuged (Remi, India) at 1,000 rpm for 10 min to remove the debris. The clear upper supernatant fluid was extracted with an equal volume of ethanol and centrifuged at 17,000 rpm for 30 min; the clear upper ethanol layer was taken and used for biochemical assay. All the preparations were performed at 4°C, and then western blotting was performed as described previously.

## Behavioral Procedures

### Open-Field Test

The effects of Drugs on the locomotors activities of the mice were evaluated automatically using an open field test with a computer-aided control system. The experiments were performed in a quiet room. The apparatus included four metal tanks (30 cm in diameter, 40 cm in height), and a video camera was fixed at the top of the device. The ceiling of the apparatus was equipped with a 120-lx light source, and four mice were tested simultaneously, each mouse was placed at the center of a metal tank and allowed to freely explore freely for 5 min. Then, locomotors activity was measured for 10 min. The total distances traveled by mice were recorded to evaluate their locomotors activities.

#### Morris Water Maze Test

##### Apparatus

The apparatus (developed by Institute of Medicinal Plant Development, Chinese Academy of Medical Sciences, and Chinese Astronaut Center, Beijing, China) is a circular water pool (100 cm in diameter and 40 cm in height) with constant clues external to the maze for spatial orientation of the mice. The water was made opaque by adding black ink to prevent animals from seeing the submerged platform. The water temperature was kept at 24– 26°C during the whole experiment. An invisible platform (6 cm in diameter and 15 cm in height) providing the only escape from water was placed 1.5 cm below the water surface. The pool was divided into four quadrants by a computerized tracking and image analyzer system. Two principal axes of the maze intersect perpendicularly to one another to create an imaginary “+.” The end of each line demarcates one of the four cardinal points: north (N), south (S), west (W), and east (E).

##### Test Procedure

MWM test was used to assess the spatial learning and memory enhancing effects of Drugs. This MWM task consisted of acquisition phase, a probe trial, and a memory retention test. On days 2–7 of behavioral measurement, spatial reference memory consisted of an acquisition phase and a probe trial, and the memory retention of the mice was tested on days 23–25.

##### Acquisition Phase

In the acquisition phase, mice were placed in the pool-containing platform to adapt to the environment before training. The platform was located in the center of the NE quadrant of the pool and remained at the same position throughout the acquisition experiment. Then mice were subjected to two trials each day for 6 days to find the submerged platform that was located in the center of the SE quadrant of the pool and remained at the same position throughout the whole experiment. Two-day training of four trials contributed to a session. For each trial, the mouse was placed for 15 s on the platform for learning; then, it was gently released into the pool facing the wall. Four different release points (NE, SE, SW, and NW) were varied randomly for each session. The mice were allowed a maximum of 180 s to find the platform. If the mouse found the platform within 180 s, it was allowed to remain there for 10 s, and its escape latency was recorded. If the mouse failed to find the platform within 180 s, it was gently guided to the platform where it remained for 10 s, and its escape latency was recorded as 180 s. Meanwhile, the swimming time spent in the target quadrant was recorded as indexes of spatial memory. After completion of daily training, the animals were returned to their cages for rest. The average of escape latency, swimming time spent in the target quadrant and swimming speed was collected to evaluate the ability of learning and memory function of mice. On the 8th day of behavioral measurement, the spatial probe trials were tested, and the platform was removed. The mice were released into the water on the opposite side of the SE quadrant. They were allowed to swim freely for 180 s. The numbers of crossings over the position at which the platform had been located, the swimming time, and the swimming distance spent in the target quadrant were recorded as indexes of spatial memory. Two weeks after MWM tests, the spatial memory retention tests were given. Neither the platform nor the starting point was fixed; mice were released in the opposite quadrant. This training had been performed two times each day for 3 days. The average of two trials during a day was determined as escape latency for the purpose of evaluating memory retention abilities of mice.

### Real-Time PCR

Total RNA was extracted from cells or tissues using Trizol Reagent (Invitrogen) according to the manufacturer’s instructions. RNA was purified by treatment with RNase-free DNase l. The concentration of total RNA was determined by a Nanodrop 2000 spectrophotometer (Thermo Fisher) at 260 nm and 280 nm. Five microgram of total RNA were reverse transcribed using the SuperScript First-Strand Synthesis System (Invitrogen). Real-time PCR was carried out in a CFX Connect PCR Detection System with SYBR Green Master Mix (Roche) and gene-specific primers. The primers were designed using the Applied Biosystems Primer Express Software (version 2.0), the specific primer sequences used for real-time PCR were as follows: for MIA40: 5’-CGGGAACAACCATGTCCTAC-3’; 5’-TCATGGTCTTCTTTGGTCACAA-3’. For KDEL receptor: 5’-ATGAATCTCTTCCGATTCCTGG-3’ and 5’-GGGAAGAAGTTGAGTTTGCCGGCA-3’. For CHOP: 5’-GCAGCTGAGTCATTGCCTTTCTC-3’; and 5’-TGCTTGGTGCAGATTCACCsATTCGG-3’. For β-actin: 5’-CACTGTGTTGGCGTACAGGT-3’; reverse: 5’-TCATCACCA TTGGCAATGAG-3’.

### Statistical Analysis

All tests were analyzed with SPSS statistical software v. 17.0 (SPSS, Inc., Illinois, Chicago, USA). For the *in vitro* studies, the results are presented as the means ± the standard deviations (SDs), and each assay was calculated from a minimum of three experiments. For the *in vivo* studies, the data are expressed as the means ± the SEMs (*n* equals the number of mice included in each analysis). One-sample Kolmogorov-Smirnov tests were used to test the normalities of the data distribution. If the data were normally distributed, statistical evaluations of the results were performed with one-way analyses of variance (ANOVAs). Multiple *post hoc* comparisons were performed using Tukey’s and the LSD test (for homogeneous variances) or the Games-Howell test (for nonhomogeneous variances). When the data distributions were not normal, the Kruskal-Wallis H test was used to analyze the differences between groups, and the differences between pairs of medians were analyzed using the Mann-Whitney U-test. The accepted level of significance for the tests was *P* < 0.05. GraphPad Prism version 5.00 (GraphPad Software, San Diego California, USA) for Windows was used to plot the data.

## Results

### STA Inhibited Aβ_25–35_-Induced Apoptosis

First, the effects of STA at different concentrations on Aβ_25–35_-treated PC12 and SH-SY5Y cells were measured using the CCK-8 assay. The results revealed that STA treatment alone (0.01–50 μM) did not alter the cell viability in PC12 (Figure 1A) and SH-SY5Y cells (Figure 1B). However, the CCK-8 assay showed that pretreatment with STA resulted in a significant reduction in Aβ_25–35_-induced toxicity, with 2 μM STA showing the strongest protective effects in PC12 (Figure 1C) and SH-SY5Y cells (Figure 1D). Furthermore, the results of the LDH release and caspase-3 activity assays confirmed the anti-apoptotic effects of STA on Aβ_25–35_-treated PC12 cells (Figures 1E,F, respectively). Again, 2 μM STA exerted the strongest neuroprotective effects. The anti-apoptotic effects of STA were further evaluated using annexin V/PI double staining and the TUNEL assay. As shown in Figures 1G,H, STA markedly reduced the number of apoptotic and TUNEL-positive cells that were induced by Aβ_25–35_. These results indicate that STA blocked the translocation of the membrane phospholipid phosphatidylserine and DNA fragmentation during Aβ_25–35_-induced apoptosis, confirming that the neuroprotective effects of STA are probably due to the inhibition of apoptotic signaling.

**Figure 1:** Santacruzamate A (STA) attenuated amyloid-β protein fragment 25–35 (Aβ_ 25–35_)-induced apoptosis and reversed Aβ_25–35_-induced unfolded protein response (UPR) and endoplasmic reticulum (ER) stress.** (A)** Effects of STA alone on the cell viability of PC12 cells. **(B)** Effects of STA alone on the cell viability of SH-SY5Y cells. **(C)** Protective effects of STA pretreatment on the Aβ_ 25–35_-induced toxicity in PC12 cells. **(D)** Protective effects of STA pretreatment on the Aβ_ 25–35_-induced toxicity in SH-SY5Y cells. **(E)** Effects of STA on lactate dehydrogenase (LDH) leakage in PC12 cells. **(F)** Effects of STA on caspase-3 activity in PC12 cells. **(G)** Effects of STA on the cell apoptosis rate in PC12 cells. Cell apoptosis was determined by annexin V/propidium iodide (PI) double staining kits using flow cytometry and quantification of the apoptosis rate. **(H)** TUNEL staining in PC12 cells. Representative images of TUNEL-positive cells (green, top row) and Hoechst counterstaining (blue, middle row) are shown, along with a histogram quantifying the TUNEL staining. Scale bar: 200 μm. This histogram shows the relative proportion of TUNEL-positive cells in different treatment groups. Cells were pre-incubated for 4 h with STA and then co-treated with Aβ_ 25–35_ for 24 h. The untreated control group was incubated with the appropriate amount of vehicle. The results are expressed as the mean ± the standard deviation of three independent experiments. ^##^*P* < 0.01 vs. the control, *P < 0.05 vs. Aβ_25–35_ treatment, **P < 0.01 vs. Aβ_25–35_ treatment.

### STA Attenuated Aβ_25–35_-Induced UPR and ER Stress

As mentioned earlier, ER stress-mediated pro-apoptotic signaling and the UPR are critical events triggered by Aβ deposition. Therefore, we assessed the levels of UPR mediators (PERK, ATF6α, and IRE1α) and ER stress markers (eIf2α, ATF4, and CHOP) to investigate whether STA affects these processes. Western blot analyses showed that pretreatment with STA for 24 h reversed the Aβ_25–35_-triggered UPR and ER stress in PC12 cells. As shown in Figure 2A, STA dramatically reversed (attenuated) the Aβ_25–35_-induced phosphorylation of PERK and IRE1α, as well as the expression of ATF6α, in PC12 cells, confirming that STA exerts effects on UPR mediators (Lin et al., 2007). As for the effects of STA pretreatment on Aβ_25–35_-induced ER stress mediators (eIf2α, ATF4 and CHOP), our analyses revealed that STA down-regulated the Aβ_25–35_-induced levels of eIF2α phosphorylation and CHOP and ATF4 expression (Figure 2B). Our findings indicate that STA blocked Aβ_25–35_-stimulated activation of the phosphorylated eIf2α–ATF4–CHOP pathway. This inhibition of the phosphorylated eIf2α–ATF4–CHOP pathway suggests that STA might reverse Aβ_25–35_-induced apoptosis by blocking the lethal ER stress-dependent pathway in PC12 cells.

**Figure 2:** STA attenuated the Aβ_ 25–35_-induced UPR and ER stress.** (A)** Effects of STA on the expression and phosphorylation of the UPR mediators PERK, ATF6α, and IRE1. **(B)** Effects of STA on the expression and phosphorylation of the ER stress markers eIf2α, ATF4, and CHOP. **(C)** Effects of STA on [Ca^2+^]_i_ overload. **(D)** Effects of STA on the levels of cleaved caspase-12. **(E)** STA reversed the Aβ_25–35_-induced Ca^2+^ current amplification. Densitometric analyses of protein bands were normalized to a loading control. Cells were pre-incubated for 4 h with STA and then co-treated with Aβ_ 25–35_ for 8 h. The untreated control group was incubated with the appropriate amount of vehicle. The results are expressed as the mean ± the standard deviation of three independent experiments. ^##^*P* < 0.01 vs. the control, **P < 0.01 vs. Aβ_25–35_ treatment.

The effects of STA on intracellular calcium ([Ca^2+^]_i_) and caspase-12 activation in Aβ_25–35_-triggered PC12 cells were also examined with the Fluo-2/AM fluorescence labeling assay. As shown in Figures 2C,D, STA reversed the Aβ_25–35_-elevated ratio of fluorescence intensity of intracellular [Ca^2+^]_i_ and the expression level of cleaved caspase-12. Moreover, patch-clamp recordings revealed that STA partly reversed the Aβ_25–35_-induced Ca^2+^ current amplification (Figure 2E). These results indicate that STA blocked the Aβ_25–35_-stimulated ER calcium release and activated the ER-mediated apoptotic pathway. Consistent with these observations, we confirmed that STA inhibited the Aβ_25–35_-induced perturbations in ER functions and prolonged UPR, which finally reversed the pro-apoptotic response.

### STA Reinforced the ER Luminal Retention of Chaperones and Activated the KDELR

To further explore the role STA plays in Aβ_25–35_-induced apoptosis, as well as the underlying subcellular mechanisms, we next investigated the effects of STA on ER-resident chaperones and the KDELR. It is known that ER chaperones are involved in a series of post-translational modifications during ER stress in the ER lumen and that they play crucial roles in preserving cellular homeostasis. The KDELR is a transmembrane protein that regulates the ER retrieval system, which takes part in the transport of ER-resident chaperones by using the C-terminal tetrapeptide KDEL motif (Ni and Lee, 2007). Western blot analyses demonstrated that STA did not alter the expression levels of the ER chaperones GRP78 and GRP94 but did elevate the expression levels of PDI and the KDELR (Figure 3A). Moreover, pretreatment with STA changed the distribution pattern of the KDELR from a point-shaped distribution to a network-like distribution (Figure 3B). The altered expression and distribution of the KDELR suggests that STA might enhance ER luminal retention of the chaperones. Therefore, we examined and detected the distribution and translocation of ER-resident chaperones in different subcellular fractions and organelles. Cross-contamination between the ER and cytosolic homogenate was slight, and the enrichment was demonstrated by using characteristic antibodies against α-tubulin and calnexin, respectively. Calnexin is an ER membrane protein that appears to be retained in the ER with no evidence of leakage into the post-ER intermediate compartment *via* the KDELR-mediated ER-retrieval system (Butler et al., 2011). Our western blot analyses showed that STA elevated the levels of GRP78, GRP94, and PDI in the ER lumen, but reduced the levels of these chaperones in the cytosol, compared with the levels in the Aβ_25–35_-treated group (Figure 3C). The immunoprecipitation assay also indicated that pretreatment with STA reversed the Aβ_25–35_-evoked dissociation of GRP78 with PERK (Figure 3D). In response to the elevated levels of misfolded proteins in the ER, GRP78 has been documented to dissociate from the ER-bound mediators of the UPR, such as PERK, and instead bind to the unfolded proteins. Hence, the reinforced binding of GRP78 to PERK that we observed indicates that STA alleviated the Aβ_25–35_-triggered UPR and ER stress. These results additionally suggest that STA reinforced ER luminal retention of the chaperones, implying that the KDELR participates in the protective effects of STA.

**Figure 3:** STA treatment up-regulated KDEL receptor (KDELR) expression, reinforced ER luminal retention of chaperones, and enhanced the binding of PERK to GRP78. **(A)** Effects of STA on the expression of GRP78, GRP94, calreticulin, protein disulfide isomerase (PDI), and the KDELR. **(B)** Pretreatment with STA changed the distribution pattern of the KDELR. Scale bar: 25 μm. Quantitative analysis of cells with altered KDELR was presented as the average data of three examined fields for different treatment group. **(C)** Effects of STA on ER luminal retention of chaperones. **(D)** Effects of STA on the binding of PERK to GRP78, as well as on the expression of the KDELR, were assessed with immunoprecipitation assays. Densitometric analyses of protein bands were normalized to a loading control. **(E)** STA reduced the levels of GRP78 and GRP94 in the mitochondria. **(F)** Effects of STA on the location of GRP78 and mitochondria, as assessed with immunofluorescent co-location assays. Scale bar: 25 μm. Quantitative analysis of colocalization was performed employing CoLocalizer Pro of CoLocalization Research Software. Background was corrected in Auto mode by selecting image pattern preset at “Average Contrast and Fluorescence.” Regions of interest (ROIs) were selected using lasso tool to include as minimum areas without fluorescence as possible. Pearson’s correlation coefficient (PCC) and an overlap coefficient according to Manders (MOCs) were examined. An average data of six examined cells were presented. Cells were pre-incubated for 4 h with STA and then co-treated with Aβ_ 25–35_ for 8 h. The untreated control group was incubated with the appropriate amount of vehicle. The results are expressed as the mean ± the standard deviation of three independent experiments. ^#^*P* < 0.05 vs. the control, ^##^*P* < 0.01 vs. the control, **P < 0.01 vs. Aβ_25–35_ treatment.

### STA Blocked ER-Resident Chaperone Translocation to the Mitochondria

As crucial factors of ER stress, ER-resident chaperones can be retargeted to the mitochondria, and thereby may be involved in correlating UPR signaling between these two organelles (Sun et al., 2006). Here, we investigated GRP78 translocation to the mitochondria by fractionating cell extracts using the mitochondrial fractionation kit and performing western blot analyses. Potential cross-contamination between the mitochondria and nuclear was ruled out using characteristic antibodies against the voltage-dependent anion channel (VDAC) and histone 2B, respectively. As expected, we observed that STA reduced the level of GRP78 in the mitochondria (Figure 3E); at the same time, immunofluorescent co-location analyses of GRP78 and mitochondria also confirmed that STA inhibited the Aβ_25–35_-induced translocation of GRP78 to the mitochondria (Figure 3F). Previous research has shown that in ER-stressed cells, GRP78 is mainly localized within the mitochondria to furnish the mitochondrial intermembrane space and matrix, thus facilitating the transmembrane transport of precursor proteins during ER stress (Malhotra and Kaufman, 2011); however, an overload of chaperones in the mitochondria may also disturb mitochondrial function (Herrmann and Riemer, 2014). Collectively, these results indicate that the STA-induced elevations in KDELR expression might be involved in attenuating the translocation of ER-resident chaperones to the mitochondria, which would contribute to the tolerance of Aβ_25–35_-triggered ER stress and concomitant activation of mitochondrial cell death pathways.

### STA Inhibited Aβ_25–35_-Induced Mitochondrial Dysfunction and Fission

Given that STA elevated KDELR expression and blocked Aβ_25–35_-induced chaperone translocation to the mitochondria, we performed a series of studies to investigate whether STA influences the structural and functional networks of the ER and mitochondria. We first detected the influence of STA on the opening of the mPTP using the calcein-cobalt quenching method. In this method, under normal conditions, calcein aggregates in the mitochondria, which is shown as areas of green fluorescence; when the mPTP opens unusually, the profound release of calcein to the cytosol is quenched by cobalt. Therefore, a reduction in the amount of green fluorescence indicates calcein-cobalt quenching and the opening of the mPTP. Furthermore, the effects of STA on Aβ_25–35_-induced MMP depolarization were visualized using the MMP-sensitive dye JC-1. JC-1 exhibits potential-dependent accumulation in the mitochondria. In normal cells, JC-1 accumulates and forms dimeric J-aggregates in the mitochondria, producing a bright red fluorescence. However, when the potential is disturbed, the dye cannot access the transmembrane space and remains in the cytoplasm in its monomer form, producing a bright green fluorescence. Consequently, mitochondrial depolarization is indicated by a reduction in the red/green fluorescence intensity ratio. As shown in Figures 4A,B, STA reversed the Aβ_25–35_ induced excessive opening of the mPTP and MMP depolarization. Subsequently, we demonstrated that STA inhibited the Aβ_25–35_-induced activation and recruitment of dynamin-related protein 1 (Drp1), mitochondrial fission protein 1 (Fis1), and mitochondrial fission factor (Mff; Figure 4C), which mediate the mitochondrial fission and apoptosis pathways. Normally, Drp1 resides in the perinuclear region of the cytosol, but during mitochondrial fission and apoptosis, Drp1 is recruited from the cytosol into the mitochondrial outer membrane, where it assembles into oligomeric complexes that entwine and compress mitochondrial tubules to facilitate fragmentation (Varadi et al., 2004; Cereghetti et al., 2008). As mitochondrial outer membrane proteins, Fis1 and Mff are required for multiple steps of Drp1-dependent mitochondrial membrane fission and serve as mediators that recruit Drp1 to the surface of the mitochondria (Lóson et al., 2013). The overexpression of Fis1 acts as a signal to promote fragmentation of the mitochondria and to facilitate the translocation of Drp1 to the mitochondrial surface during recruitment (Stojanovski et al., 2004). Mff is another critical factor in Drp1 recruitment and functions as an essential receptor to stimulate Drp1-mediated mitochondrial fission (Otera et al., 2010). The effects of STA that we observed on these factors indicate that STA can reverse Aβ_25–35_-triggered mitochondrial dysfunction and structural fission.

**Figure 4:** STA inhibited the Aβ_25–35_-induced mitochondrial fission and apoptosis pathways, and the KDELR contributed to the cytoprotective effects of STA. **(A)** Effects of STA on the opening of the mitochondrial permeability transition pore (mPTP), as assessed using the calcein-cobalt quenching method. After treatment(s), cells were loaded with calcein dye and incubated with cobalt chloride, the emission wavelengths of which were 488 and 505 nm, respectively. The mPTP of cells in each group was calculated by examining the level of green fluorescence and analyzed using a fluorescence microplate reader. Scale bar: 100 μm. **(B)** The effects of STA on Aβ_25–35_-induced mitochondrial membrane potential (MMP) depolarization were visualized using the MMP-sensitive dye JC-1. Red fluorescence from JC-1 indicates healthy mitochondria with polarized inner mitochondrial membranes, while green fluorescence is emitted by cytosolic JC-1 monomers and indicates MMP dissipation. Merged images indicate the co-localization of JC-1 aggregates and monomers. The MMP was analyzed using a fluorescence microplate reader after JC-1 staining. Scale bar: 50 μm. The results are expressed as a percentage of the control. **(C)** Effects of STA on the levels of Drp1, Fis1, and Mff in the mitochondrial fraction. **(D)** Effects of STA on the levels of mitochondrial intermembrane space assembly protein 40 (Mia40), ALR, Tom40, and Tim23. **(E)** Effects of STA on the levels of cleaved caspase-9, released cytochrome C, Smac, and AIF. **(F)** KDELR knockdown abolished the STA-alleviated ER stress and apoptosis. **(G)** KDELR knockdown abrogated the STA-reversed retention of ER chaperones and ER stress. **(H)** KDELR knockdown attenuated the anti-apoptotic effects of STA. **(I)** KDELR knockdown reversed the effects of STA on [Ca^2+^]_i_. Densitometric analyses of protein bands were normalized to a loading control. Cells were pre-incubated for 4 h with STA and then co-treated with Aβ_ 25–35_ for 8 h (24 h in H). The untreated control group was incubated with the appropriate amount of vehicle. The results are expressed as the mean ± the standard deviation of three independent experiments. ^#^*P* < 0.05 vs. the control, ^##^*P* < 0.01 vs. the control, *P < 0.05 vs. Aβ_25–35_ treatment, **P < 0.01 vs. Aβ_25–35_ treatment.

### STA Reversed the Mitochondrial Intermembrane Space Assembly Pathway

As the cell’s powerhouses, the mitochondria play crucial roles in integrating pro-apoptotic signals during harmful ER stress (Malhotra and Kaufman, 2011). This, coupled with the above results, indicate that the STA-triggered inhibition of ER-resident chaperone translocation to the mitochondria might restore the Aβ_25–35_-triggered mitochondrial dysfunction and inhibit the Aβ_25–35_-triggered activation of the fission and apoptosis pathways. To gain deeper insight into the mechanisms of this process, we analyzed mitochondrial transmembrane transport during chaperone translocation. As shown in Figure 4D, STA reversed the reductions in Mia40-ALR that were induced by Aβ_25–35_, while the expression levels of the translocase of the mitochondrial outer membrane protein 40 (Tom40) and translocase of the inner mitochondrial membrane protein 23 (Tim23) were not noticeably influenced. During protein synthesis in the cytosol, the mitochondrial intermembrane space assembly pathway plays a significant role in the transmembrane transport of mitochondrial proteins. Cytosolic proteins are specifically recognized by the Mia40 protein and are oxidized through the cooperative action of Mia40 and ALR/Erv1. Mia40 functions as a receptor, folding catalyst, and disulfide carrier, while the ALR protein serves as a sulfhydryl oxidase. Moreover, COX6B and COX17 are the substrate proteins recognized by Mia40 (Bragoszewski et al., 2015). Hence, the present results imply that pretreatment with STA also attenuated the levels of COX6B and COX17 compared with the Aβ_25–35_-treated group (Figure 4E). Our observations suggest that STA might mitigate the effects of Aβ_25–35_ on Mia40-ALR through blocking chaperone translocation to the mitochondria. Furthermore, STA attenuated the Aβ_25–35_-induced up-regulation of cleaved caspase-3 and blocked the Aβ_25–35_-induced up-regulation of released cytochrome C, Smac, and AIF (Figure 4F). These results suggest that STA might suppress Aβ_25–35_-related activation of the mitochondrial fission and apoptosis pathways by reversing the mitochondrial intermembrane space assembly pathway, potentially by increasing KDELR expression and blocking chaperone translocation to the mitochondria.

### The KDELR Contributed to the Cytoprotective Effects of STA on Aβ_25–35_-Induced Apoptosis

To confirm the positive role of the KDELR in the STA-generated anti-apoptotic effects that were noted above, we knocked down the KDELR with small interfering RNA (siRNA). As shown in Figures 4G,H, the KDELR knockdown demonstrated significantly attenuated the STA-induced cytoprotection, elevated levels of phosphorylated-PERK, and reduced expression of GRP78 in the ER lumen compared with the wild-type (WT) group. Furthermore, knocking down the KDELR also reversed the STA-mediated recovery of [Ca^2+^]_i_ homeostasis (Figure 4I), suggesting that the KDELR might play a crucial role in ER-resident chaperone translocation to the mitochondria, which might eventually counteract Aβ_25–35_-induced ER stress and the associated activation of the mitochondrial cell death pathway.

### Effects of STA on Mouse Locomotive Activities in the Open-Field Test

To confirm whether STA might be a promising agent for treating the cognitive deficits of AD, we evaluated the effects of STA on the learning and memory impairments in the APPswe/PS1dE9 transgenic mouse model of AD using the open-field, MWM, and step-down passive avoidance tests. The animal treatments and behavioral test procedures are described in the supporting information and are presented in Figure 5A. At first, no significant effects of STA (5 and 10 mg/kg) on mouse locomotive activities in the open-field test were observed in the APPswe/PS1dE9 group compared with the WT group (Figure 5B).

**Figure 5:** Behavioral tests. **(A)** Experimental procedure. **(B)** Locomotive activities in the open-field test. In acquisition trials of the Morris water maze (MWM), training trials were performed on days 2–7 to measure the **(C)** escape latency, **(D)** swimming time spent in the target quadrant, and **(E)** swimming speed. The probe trial was performed 24 h after the acquisition tests to measure the **(F)** crossing numbers, **(G)** swimming time spent in the target quadrant, and **(H)** swimming speed. The memory retention tests were conducted on days 23–25 of the behavioral tests to measure the **(I)** escape latency, **(J)** swimming time spent in the target quadrant, and **(K)** swimming speed. The results are expressed as the mean ± the standard deviation of three independent experiments. ^#^*P* < 0.05 vs. the control, ^##^*P* < 0.01 vs. the control, *P < 0.05 vs. Aβ_25–35_ treatment, **P < 0.01 vs. Aβ_25–35_ treatment.

### Effects of STA on APPswe/PS1dE9 Mice in the MWM Test

In the acquisition trials, short escape latencies and large percentages of time spent in the target quadrant were observed over the course of the training trials in all groups (Figures 5C,D), indicating that regardless of the treatment applied, the learning and memory functions of mice improved over the course of training. As expected, a significant difference was observed in the escape latency and percentage of time spent in the target quadrant between the WT and APPswe/PS1dE9 groups in sessions 2 and 3 (Figures 5C,D). The results indicated that APPswe/PS1dE9 mice took longer to locate the platform than did WT mice, likely owing to deterioration of their spatial memory ability. By contrast, STA notably shortened the escape latency and increased the percentage of time spent in the target quadrant in sessions 2 and 3 (Figures 5C,D). The shortened escape latencies and increased escape rates implied that STA attenuated the spatial learning deficits in APPswe/PS1dE9 mice. Meanwhile, no significant differences in swimming speed were noted among the groups across all of the training trials (Figure 5E), and hence the observed improvements in memory and learning that were induced by STA were likely not related to changes in the swimming speed.

In the spatial probe trials, the number of crossings was significantly lower in APPswe/PS1dE9 mice than in WT mice, while STA markedly elevated the number of crossings (Figure 5F). Additionally, the shorter swimming time in the target quadrant in APPswe/PS1dE9 mice was significantly reversed by STA (Figure 5G). It should be noted that STA treatment permitted the APPswe/PS1dE9 mice to form a memory of the platform location. Meanwhile, the swimming speed was not significantly different among the groups during the probe trials (Figure 5H), which again supports that the effects of STA are not related to changes in swimming speed and/or physical strength.

In the memory retention tests, APPswe/PS1dE9 mice demonstrated a much longer escape latency and smaller percentage of time spent in the target quadrant than did WT mice in all three sessions (Figures 5I,J). By contrast, APPswe/PS1dE9 mice treated with different concentrations of STA demonstrated a dramatically reduced escape latency and a larger percentage of time spent in the target quadrant. As above, the swimming speed did not significantly differ among the groups during the memory retention tests (Figure 5K). These results indicate that STA ameliorated the memory deficits in APPswe/PS1dE9 mice to a certain extent and that the improvements were not related to changes in swimming speed.

### Effects of STA on the KDELR and Mia40 in the Brain Tissue of Mice

To investigate the possible neuropathological correlates of the STA-activated KDELR and Mia40-ALR functions, as well as associative memory, in APPswe/PS1dE9 transgenic mice, immunohistochemical and immunoblot analyses of the brain tissue of each mouse group were performed after completion of the behavioral studies. As shown in Figures 6A,B, immunoblot data confirmed that STA enhanced the expression levels of KDELR and Mia40, while the RT-PCR analyses revealed that STA only enhanced the transcription levels of KDELR, not Mia40, in the brain tissue of APPswe/PS1dE9 mice. Such findings imply that the STA-induced up-regulation of Mia40 might be due to the reduced degradation of Mia40. These results confirm that STA attenuated harmful ER stress in the hippocampus of APPswe/PS1dE9 mice and suggest that the STA-enhanced KDELR and Mia40-ALR functions might be involved in ameliorating the cognitive deficits and memory impairments that are associated with AD (Figure 6C).

**Figure 6:** Biochemical evaluation of brain tissue. **(A)** Immunoblot analysis of CHOP, KDELR, and Mia40. **(B)** RT-PCR analysis of CHOP, KDELR, and Mia40. **(C)** Schematic diagrams delineating the STA inhibited Aβ_25–35_-induced UPR and ER stress by regulating the KDELR, which reinforced the retention of resident chaperones and blocked Aβ_25–35_-induced ER chaperone translocation to the mitochondria and restored the Mia40-ALR system, ultimately attenuating the Aβ_25–35_-induced apoptosis pathways. Densitometric analyses of protein bands were normalized to a loading control. The results are expressed as the mean ± the standard deviation of three independent experiments. ^##^*P* < 0.01 vs. the control, *P < 0.05 vs. Aβ_25–35_ treatment, **P < 0.01 vs. Aβ_25–35_ treatment.

## Discussion

The present study demonstrated the neuroprotective effects of STA, a carbamate derivative, against Aβ_25–35_-induced toxicity, as well as the relevant molecular mechanisms. We also confirmed that STA was effective in promoting memory performance in APPswe/PS1dE9 mice. Together, our data support that STA has the potential to ameliorate AD-like pathology and reverse the associated cognitive deficits by attenuating pathological changes and neuron lesions.

Herein, we first confirmed the anti-apoptotic effects of STA and revealed that STA ameliorated the Aβ_25–35_-triggered UPR and ER stress. In addition, we demonstrated that STA altered the intracellular trafficking of ER-retained chaperones, thus causing an elevation in ER chaperone retention. As a neurotoxin, Aβ_25–35_-induced ER stress is involved in the assembly of newly synthesized or misfolded proteins during the UPR in the ER lumen (Viana et al., 2011), which plays crucial roles in preserving cellular homeostasis (Eletto et al., 2010). Furthermore, our observations highlighted the significant role of the KDELR-mediated ER-retrieval system in Aβ_25–35_-induced ER stress (Capitani and Sallese, 2009). It is known that ER chaperones contain a carboxyl-terminal retrieval signal, namely the KDEL (Lys-Asp-Glu-Leu) sequence, which is recognized by the KDELR; the KDELR then facilitates the retrograde transport of chaperones from the post-ER compartment (Cancino et al., 2013). Retro-transport of these chaperones encourages the retrieval and return of misfolded proteins to the ER for refolding or ER-associated degradation, thus regulating ER quality (Smith et al., 2011). However, the extensively sustained induction of ER chaperones and cargo loading may saturate KDELR-mediated retrieval and modify the expression and distribution of the KDELR (Li et al., 2015). When KDELR-mediated retrieval is limited, a number of newly synthesized ER-retained chaperones, such as the heat shock protein family including GRP78, GRP94 and other co-chaperones like folding enzymes PDI, may avoid retrieval and exit the ER lumen, dramatically aggravating ER stress (Ni and Lee, 2007). Our data indicated that STA might enhance ER luminal retention of the chaperones and ER stress tolerance *via* regulating the KDELR.

The present study additionally demonstrated that STA blocked GRP78 translocation to the mitochondria and reversed the concomitant mitochondrial dysfunction and fission. Normally, GRP78 is located in the ER lumen to the post-ER compartment but would translocate to the mitochondria from the ER, thus counteracting the ER stress-triggered apoptotic signals and responses (Sun et al., 2006). In the present study, the Aβ_25–35_-induced ER-resident chaperone translocation to the mitochondria seemed to be positively associated with the abnormal opening of the mPTP, MMP depolarization, and recruitment of Drp1-dependent mitochondrial membrane fission, which established a link between chaperone translocation to the mitochondria and apoptosis. Importantly, our findings suggest that STA might reverse Aβ_25–35_-triggered mitochondrial dysfunction by restoring the mitochondrial intermembrane space assembly pathway and Mia40-ALR system. Since most mitochondrial proteins originate in the cytosol, mitochondria have developed an import and retrograde system to maintain the equilibrium of transmembrane transport (Fan and Young, 2011; Ceh-Pavia et al., 2013). The mitochondrial intermembrane space assembly pathway mediates the folding and redox-dependent import of precursor proteins (Bragoszewski et al., 2015), with Mia40 and ALR being responsible for mediating the oxidative folding of proteins (Neal et al., 2015). When cytosolic proteins enter the Tom complex channel, Mia40 specifically recognizes precursor proteins and serves as a receptor and oxidoreductase (Wiedemann et al., 2004); meanwhile, ALR serves as a sulfhydryl oxidase. Following this, Mia40-mediated proteins are translocated across the inner mitochondrial membrane and transferred to the matrix *via* the Tim complex (Wrobel et al., 2013). Interestingly, Aβ_25–35_ attenuated the Mia40-ALR levels, and induced an accumulation of their substrate proteins, COX6B and COX17. These observations suggested that the Aβ_25–35_-triggered trafficking of chaperones might be associated with mitochondrial transmembrane transport. Significantly, STA increased the levels of Mia40-ALR and blocked the translocation of mitochondrial intermembrane space proteins. Therefore, we hypothesize that chaperone translocation to the mitochondria from the ER might occur in order to harmonize UPR signaling between the two organelles; however, the overload of GRP78 translocation may act as a harmful event during Aβ_25–35_-induced ER stress and mitochondrial dysfunction.

From the above results, it is conceivable that proper temporospatial controls of molecular chaperones are important for influencing their functions during ER stress and the UPR and as shown in the Figure 6, the STA-induced regulation of the KDELR may be crucially involved in chaperone trafficking, thus ameliorating Aβ_25–35_-induced pro-apoptotic cascades. Importantly, our behavioral results and biochemical evaluations in brain tissue were consistent with the results of our *in vitro* experiments and support the essential role the KDELR plays in ameliorating memory impairment. It is worth noting that STA enhanced the transcriptional levels of the KDELR, but not of the Mia40 protein. Therefore, we speculate that STA ameliorated the memory impairments in the AD mouse model by intervening in the transcriptional regulation of the KDELR. Additionally, the affected Mia40 might be due to the attenuation of the degradation and depletion.

In conclusion, our study not only confirmed that STA was able to effectively attenuate Aβ_25–35_-induced toxicity and promote memory performance in APPswe/PS1dE9 mice but also provided potential evidence of the underlying mechanisms. Our data suggest that Mia40-ALR and the KDELR might be activated synergistic targets that mediate ER stress tolerance and support that carbamate derivatives may be promising agents for reversing the progression of AD. STA in particular appears to be a potential candidate compound for treating ER stress- and UPR-related neurodegenerative disorders.

## Author Contributions

WLi and ZL designed the experiment and wrote the article. LC and YL performed the experiment. HT, YZ and JX processed the data.WLiu revised the article.

## Conflict of Interest Statement

The authors declare that the research was conducted in the absence of any commercial or financial relationships that could be construed as a potential conflict of interest.
